This article has been retracted.

# A 3D-2D Convolutional Neural Network and Transfer Learning for Hyperspectral Image Classification

**DOI:** 10.1155/2021/1759111

**Published:** 2021-08-21

**Authors:** Douglas Omwenga Nyabuga, Jinling Song, Guohua Liu, Michael Adjeisah

**Affiliations:** ^1^School of Computer Science and Technology, Donghua University, Shanghai, China; ^2^School of Mathematics and Information Technology, Hebei Normal University of Science & Technology, Qinhuangdao, Hebei, China

## Abstract

As one of the fast evolution of remote sensing and spectral imagery techniques, hyperspectral image (HSI) classification has attracted considerable attention in various fields, including land survey, resource monitoring, and among others. Nonetheless, due to a lack of distinctiveness in the hyperspectral pixels of separate classes, there is a recurrent inseparability obstacle in the primary space. Additionally, an open challenge stems from examining efficient techniques that can speedily classify and interpret the spectral-spatial data bands within a more precise computational time. Hence, in this work, we propose a 3D-2D convolutional neural network and transfer learning model where the early layers of the model exploit 3D convolutions to modeling spectral-spatial information. On top of it are 2D convolutional layers to handle semantic abstraction mainly. Toward simplicity and a highly modularized network for image classification, we leverage the ResNeXt-50 block for our model. Furthermore, improving the separability among classes and balance of the interclass and intraclass criteria, we engaged principal component analysis (PCA) for the best orthogonal vectors for representing information from HSIs before feeding to the network. The experimental result shows that our model can efficiently improve the hyperspectral imagery classification, including an instantaneous representation of the spectral-spatial information. Our model evaluation on five publicly available hyperspectral datasets, Indian Pines (IP), Pavia University Scene (PU), Salinas Scene (SA), Botswana (BS), and Kennedy Space Center (KSC), was performed with a high classification accuracy of 99.85%, 99.98%, 100%, 99.82%, and 99.71%, respectively. Quantitative results demonstrated that it outperformed several state-of-the-arts (SOTA), deep neural network-based approaches, and standard classifiers. Thus, it has provided more insight into hyperspectral image classification.

## 1. Introduction

Hyperspectral images (HSIs) have hundreds of spectral bands that comprise detailed spectral information. As a result, HSI images have formed the foundation for a wide range of applications, including precision agriculture [1], resource surveys [2], target identification [3], and landscape classification [4]. Because visual classification can aid in interpreting HSI image scenes, classification is an essential domain in HSI image processing [5, 6]. However, high dimensionality, high nonlinearity, and an imbalance between the limited training samples of HSIs [7, 8] affect classification accuracy and make HSI classification difficult.

To address the abovementioned challenges, dimensionality reduction (DR) [9–12] and semisupervised classification [13, 14] approaches have been extensively adopted for HSIs. Generally, there are two classes of DR, i.e., the band selection and feature extraction [15]. Among them, feature extraction [16–19] minimizes computational complexity by projecting high-dimensional data into low-dimensional data space and feature selection [20] picks appropriate bands from the original set of spectral bands. Further, a sparse-based method [21] has been used to derive useful spectral features. Nevertheless, PCA seeks out the best orthogonal vectors for representing information from HSIs [22, 23] with minimized spectral dimension (up to 85%). On the contrary, it improves the separability among classes, decreases, and brings a balance of the interclass and intraclass. Therefore, we used PCA as an effective tool to transform the original features into a new space with reduced dimensionality and more excellent distinctive features.

Lately, a more innumerable center has been directed to the remote sensing (RS) study scope for HSI classification. However, the high-resolution features of HSI data make it challenging to understand and separate several land-cover classes, extract more major distinctive structures, and produce an unbiased HSI classification through the application of traditional machine learning (ML) approaches [24]. Nonetheless, the evolution of deep learning (DL) has exceptionally improved not only in RS but also in different research areas such as digital image processing (DIP), pattern recognition, segmentation, data classification, and object detection [25]. The tremendous progress in DL to analyze HSI [26] by many research works in the past years has somewhat solved the HSI classification problem through a proposed dual-path network (DPN). It combined two systems, specifically the dense-convolutional network and the residual network [27]. It engages an unsupervised greedy layer-wise training approach to interpret the RS images [28] for a pixel-block pair (PBP) exhibition. To find a solution for HSI classification, Song et al. [29] came up with a deep feature fusion network while Cheng et al. [30] adopted the off-the-shelf convolutional neural network (CNN) techniques. Li et al. [31] employed 3D-CNN, deep feature extraction for HSI classification. Mou et al. [32] considered an unsupervised model referred to as a deep residual conv-deconv network to resolve the HSI classification problem.

However, the rarity of identifying the HSI pixels of the separable classes is a repeated integrated obstacle in the original space. It is patent from this past research that singularly employing 2D-CNN or 3D-CNN has limitations, for instance, squandered band-related information or deeply intricate method. Additionally, it prevents the methods mentioned above from achieving outstanding accuracy. The principal explanation is that HSI is volumetric data with spectral dimension. Using the 2D-CNN method alone cannot acquire helpful, distinctive feature maps from the spectral interpretations. Likewise, a deep 3D-CNN method is computationally costly. It performs poorly for classes of similar features over several spectral channels when used alone. In addition, the methods take more computational time to analyze and interpret the spectral-spatial data cubes.

Therefore, we proposed a 3D-2D convolutional neural network and transfer learning model embedded in ResNeXt-50 with consecutive feature learning blocks based on the challenges mentioned above. Our approach takes the spectral-spatial features of HSI into account for classification. It achieves a brief description of the spectral-spatial data and enhanced computational efficiency as defined:

  We propose a 3D-2D convolutional neural network and transfer learning model that utilizes 3D convolutions to modeling spectral-spatial information in the early network layers of the model and the 2D convolutions on top to exceptionally deal with semantic abstraction.
  The network leverage convolutional blocks of the ResNeXt-50 model before the flatten layer to further enhance the performance.
  We applied regularization techniques to avoid overfitting during fine-tuning. We engaged an optimizer with a prolonged learning rate with a dropout of 0.5/0.055 and early stopping in the training process. Adam is a good choice for the process as opposed to methods such as stochastic gradient descent (SGD).
  We evaluated our proposed model on five sets of publicly available HSI data. Our proposed model delivers swift spectral-spatial representation, enhances computational efficiency, and validates more understanding of the 3D spectral-spatial hyperspectral imagery classification.

The rest of our paper is organized as follows; Section 2 gives the related works on HSI classification. Then, Section 3 describes the proposed approach in detail.  Section 4 presents extensive experiment; finally, the conclusion is presented in Section 5.

## 2. Related Work

Recently, CNNs have been implemented by a manifold of researchers; for example, Zhang et al. [33, 34] implemented a CNN model for the HSI classification. The work acquired the spatial features through a 2D-CNN approach by utilizing the original HSI image's first insufficient principal component channels. Using 2D-CNN in HSI comes with various advantages: a principled way to acquire features instantly from the original input images. It has shown tremendous promise in image processing and computer vision, with applications such as object detection [35] and image classification [36]. Nonetheless, the immediate deployment of 2D-CNN to HSI images necessitates the convolution of individual inputs of the 2D networks, in addition to each group of learnable kernels. Frequently, a substantial amount of bands with the spectral dimension of the HSI image requires a vital number of parameters, which may be subject to overfitting and a risen computational cost.

Preceding articles acknowledge that 2D-CNN has achieved incredible outcomes in visual data processing areas such as image classification [37], face detection [38], depth estimation [35, 39], and object detection [40]. Nevertheless, using 2D-CNN in the investigation of HSI points to the failure to catch channel-related information. Accordingly, using 2D-CNN entirely has no capacity for extracting valuable features of the spectral dimension. In addition, the 2D-CNNs, when deployed alone, hinder them from achieving more reliable accuracy on HSI.

An enhanced spatial dimension of HSIs helps supply multiple low-level features, combining exhaustive spatial information. In contrast, the spectral features present fundamental and distinguishing features to reveal the components of land objects [41]. Hence, the deployment of spectral-spatial information advances and increases HSI classification efficiency. The 3D-CNN [42] model proposed by Ben Hamida et al. focused on exploring different DL techniques for HSI dataset classification. Zhong et al. [43] implemented a 3D deep learning framework for spectral-spatial features classification. To extract the spatial-spectral features undeviatingly from the original HSI image, Mei et al. [44], introduced a 3D CNNs approach that exhibited boosting classification outcomes. Li et al. [45] extended their investigations of 3D-CNN to classify spectral-spatial with the use of 3D input cubes with small spatial dimensions. Their techniques produce thematic classification maps employing an approach that can process original HSIs directly. However, the CNN method drops in precision as the network deepens.

Li et al. [46] further explain that HSI imagery combines several adjacent bands or channels with affluence of spectral signatures, hence, the distinguishing of different elements through discrete spectral discrepancies. However, these spectral bands are closely correlated and incorporate considerable redundant information due to a huge volume of the raw spectral bands and the spatial resolution, henceforward, the difficulty in discriminating the land-cover classes [47]. Additionally, the key enigma entails extracting the discriminative features of the HSI data to reduce the set of important bands [48]. In a different outline, the HSI data generally takes a 3D cube form. The 3D convolution in spectral-spatial dimensions frequently contributes towards an effective approach that empowers a concurrent extraction of the detailed features in such images. Studying the information, numerous authors have implemented a 3D-CNN method to purposely extract the deep spectral-spatial [18, 30, 36, 42, 43, 45, 49, 50]. Works by Song et al. [29], Mou et al. [32], Zhong et al. [43], and Paoletti et al. [51] exhibited extensive network residual learning (RL) models to extract additional discriminative characteristics for HSI classification. More advanced investigations on HSI classification point to significant enhancement by fusing spatial features toward classifiers [52]. Although the 3D-CNN architectures are manageable and can deduce the spectral and spatial information from HSI data while accomplishing more reliable accuracy, they are computationally expensive to be uniquely employed in HSI analysis. On the contrary, when deployed alone, it hinders them from achieving more reliable accuracy on HSIs. It is essential to merge the learned spatial features with the spectral features captured by feature extraction methods for reliable HSI classification.

Melgani and Bruzzone [53] introduced a support vector machine (SVM) technique with diverse classifiers to evaluate their potentials. Makantasis et al. [19] proposed deep learning that envisions high-level features automatically in a hierarchical order to encode spatial information and pixels' spectral for classification. They engaged a 3D DL method that facilitated spectral and spatial information and then induced a basis for solving RS data noise. The method subsequently classified the information employing a multilayer perceptron. However, the method only considered spatial features for HSI classification. A multiscale 3D deep CNN (M3D-DCNN) of 5 layers is proposed for similar work [54]. The model concurrently learns 2D multiscale spatial features and 1D spectral features from HSI data in an end-to-end approach. Thus, it jointly extracts both the multiscale spatial feature and the spectral feature. Moreover, the model lacks features aggregation, which affected classification performance.

Zhong et al. built a spectral-spatial residual network (SSRN) model that manipulates the 3D raw data cubes for HSI classification [43]. It uses identity mapping to concatenate 3D convolutional layers via residual blocks for backpropagated gradients. Using hybrid spectral CNN (HybridSN), Roy et al. [55] achieved a better classification accuracy. The model combines the corresponding spectral and spatio-spectral data in the 3D and 2D convolution forms, respectively. Although the model achieved high accuracy, it maintains many parameters likened to the SSRN model; simultaneously, it takes a long to train.

In this context, our system shares the same skeleton system architecture as Roy et al. [55], except for the convolved 2D input kernels. Instead of a single 2D layer, we leverage five (5) convolutional blocks of the ResNeXt-50 model starting from the layer block with filter 128 before the flatten layer to handle semantic abstraction. We freeze the layers from the 3rd block before training. This practice strongly discriminates the spatial information within different spectral bands without substantial loss of spectral information. The experimental result shows that the approach improves the computational efficiency, classification accuracy, and instantaneous representation of the spectral-spatial information compared to SOTA methods such as SVM [53], 2D-CNN [19], 3D-CNN [42], M3D-CNN [54], SSRN [43], and HybridSN [55] that have deployed the hyperspectral remote sensing images as the experimental datasets.

## 3. Proposed Method

### 3.1. A 3D-2D Convolutional Neural Network and Transfer Learning Model

Figure 1 illustrates the general diagram of our proposed method for hyperspectral image classification.

The proposed 3D-2D convolutional neural network and transfer learning model (3D-2D-CNNTL) model mimics the design architecture of HybridSN but differs in implementation. It fuses both 3D and 2D-CNN layers to obtain the spectral features encoded in a manifold of bands with spatial information. The 3D-CNN learns an abstract level spectral-spatial representation and the 2D-CNN network for spatial feature learning. We then leverage convolutional blocks of the ResNeXt-50 model before layer flatten. ResNeXt-50 blocks are deep residual networks with cardinality that utilizes the split-transform-merge method. Results are seen in branching paths within a cell to transform the residual block. The output from the ResNeXt-50 block concatenated with the skip connection path resulting in an orthogonal increase in the depth of the residual networks [56]. The ResNeXt-50 block is represented as

(1) $$\begin{array}{c} y=x+\sum_{i=1}^{C}\tau_{i}\left(x\right), \end{array}$$

where *y* is the output, *x* represents the input of the preceding network layer, *C* denotes the cardinality, and *τ*_*i*_ is the arbitrary function that projects *x* into low-dimensional embedding and transforming it. The proposed model network concatenated with ResNeXt-50 as the base model is shown in Figure 2.

### 3.2. Hyperspectral Input Image

As shown in equation (2), we took the input image as the spectral-spatial hyperspectral data cube represented by

(2) $$\begin{array}{c} I\in R^{W\times H\times N}, \end{array}$$

where **I** denotes the HSI input image, *W* denotes the width, while *H* denotes the height, and *N* signifies the value of spectral bands. Each spectral-spatial image pixel in **I** consist of *N* spectral measures which formulate to a label vector expressed as

(3) $$\begin{array}{c} \bar{V}=\left(v_{1},v_{2},\ldots ,v_{C}\right)\in R^{1\times 1\times L}, \end{array}$$

where *L* in this space represents the land-cover categories.

### 3.3. Dimensionality Reduction

PCA is an unsupervised feature technique for feature extraction used to derive orthogonal features from a dataset and decrease the feature space's dimensionality. We applied PCA for dimensionality reduction at the first **I**, beside the spectral channels, to eliminate spectral redundancy and dataset imbalance. This redundancy is caused by high intraclass variability and interclass similarity due to different land-cover classes represented by the spectral-spatial HSI pixel. To identify the object in its original class, the PCA helps to decrease spectral bands, i.e., from *N* to *S* but conserved *W* and height *H* at the exact spatial dimensions, as shown in the equation below:

(4) $$\begin{array}{c} P\in R^{W\times H\times N}, \end{array}$$

where **P** denotes the transformed HSI input after applying PCA. We then divided the spectral-spatial data cubes into small overlapping 3D patches *Q* ∈ *R*^*S*×*S*×*N*^ from **P**, where *S* × *S* represents the width and height of the covering window size. Finally, the central pixel of the class label at the spatial location (*α*, *β*) decides the truth labels. The 3D patches (*n*) from *S* takes expression

(5) $$\begin{array}{c} \left(W-S+1\right)\times \left(H-S+1\right). \end{array}$$

The 3D patch at the position (*α*, *β*), represented by *Q*_(*α*, *β*)_, thus represents the width from (*α* − (*S* − 1)/2) to (*α*+(*S* − 1)/2), height with the entire *N* spectral bands of PCA decomposed data cubes **P**.  Figure 3 delineates the process of dimensionality reduction.

There are four primary steps in PCA as the pseudocode for each computing step is supplied in Algorithm 1. The data volume is first relocated to a new location to be recentered around the reference origin region. The mean value of each spectral band is computed and removed during data preprocessing (see step 2 of Algorithm 1). Second, the data volume's covariance matrix is calculated as the product of the preprocessed data matrix and its transpose (step 3). The related eigenvectors of the covariance matrix are then retrieved (step 4). Each pixel of the original image is projected into a subset of eigenvectors (steps 5 and 6), which produce a reduced dimensionality.

We can get a reduced dataset from the original high-dimensional dataset by following these steps, which is the primary goal of the PCA technique. Finally, the explained variance ratio given by a principal component is the balance between the variance of that principal component and the total variance. The explained variance ratio was nearly 75% for the five dataset samples.

### 3.4. The Spectral-Spatial Feature Learning

To generate the feature maps of the convolution layer from the spectral-spatial features and capture the spectral information, we applied the 3D kernel over a manifold of adjacent HSI channels in the input layer in our suggested model for the HSI dataset. The 3D convolution network at a spatial point (*x*, *y*, *z*), which denotes the activation value at the *j*^th^ feature map of the *i*^th^ network layer of the proposed model, is designated as *v*_*i*,*j*_^*x*,*y*,*z*^ and produced through the following expression:

(6) $$\begin{array}{c} v_{i,j}^{x,y,z}=\phi \left(b_{i,j}+\sum_{r-1}^{d_{l-1}}\sum_{\lambda =-\eta }^{\eta }\sum_{\rho =-\gamma }^{\gamma }\sum_{\sigma =-\delta }^{\delta }w_{i,j,\tau }^{\sigma ,\rho ,\lambda }\times v_{i-1,\tau }^{x+\sigma ,y+\rho ,z+\lambda }\right), \end{array}$$

where *ϕ* represents the activation function, the bias constraint is denoted by *b*_*i*,*j*_, *d*_*l*−1_ signifies the value of feature map in *l* − 1^th^ network layer, 2*γ*+1 represents kernel's width, 2*δ*+1 is the height of kernel, the depth of the kernel is represented by 2*η*+1 along the spectral dimension, and *w*_*i*,*j*_ represents the number of weight constraint of *i*^th^ network layer for the *j*^th^ feature map.

We applied a supervised approach [36] to train the constraints of bias represented by (*b*) and the kernel weight represented by (*w*) through gradient descent. Eventually, a spectral-spatial feature representation is taken concurrently from the HSI by the 3-D-CNN kernel, whereby the computational expense remains complex. To achieve the convolution of the network, we estimated the summation of products of the two corresponding dot products. These products are the HSI input and the kernel spatial dimensions. Lastly, we include the entire feature maps of the last network layer of the model. The activation function value in 2D convolution at (*x*, *y*) denotes the spatial point of the *i*^th^ network layer for the *j*^th^ feature map represented by *v*_*i*,*j*_^*x*,*y*^ and generated using the in-text equation:

(7) $$\begin{array}{c} v_{i,j}^{x,y}=\phi \left(b_{i,j}+\sum_{r-1}^{d_{l-1}}\sum_{\rho =-\gamma }^{\gamma }\sum_{\sigma =-\delta }^{\delta }w_{i,j}^{\sigma ,\rho }\times v_{i-1,\tau }^{x+\sigma ,y+\rho }\right), \end{array}$$

where *ϕ* in the equation represents the activation function, *b*_*i*,*j*_ denotes bias constraint, *d*_*j*−1_ signifies the value of feature map in *l* − 1^th^ network layer, and *w*_*i*,*j*_ represents the width of the kernel all designed for the *i*^th^ network layers for the *j*^th^ feature maps.

A 3D convolution is produced via concatenating a 3D kernel with 3D data. Roy et al. [55] employed a 3D kernel over a manifold of adjoining bands and channels in the input layer to obtain the spectral features to generate a feature map layer. We employed similar 3D for the first three layers in our model. Triple 3D convolutions (Conv3D) are applied to preserve the spectral features for the input data. This helps the amount of spectral-spatial (SS) feature maps to increase within the output dimensions simultaneously. We engaged 3D convolutional blocks with filters; 8, 16, and 32 in the first, second, and third convolution layers. The Conv3D and Max-Pooling kernel size is *z* × *z* × *h*, that is, *z*= kernel spatial size and *h*= the kernel depth. Conv_layer1 = 8 × 3 × 3 × 7(Ζ_1_^1^=3, Ζ_2_^1^=3, Ζ_3_^1^=7), Conv_layer 2 = 16 × 1 × 1 × 1(Ζ_1_^2^=1, Ζ_2_^2^=1, Ζ_3_^2^=1), and Conv_layer3 = 32 × 1 × 1 × 1(Ζ_1_^3^=1, Ζ_2_^3^=1, Ζ_3_^3^=1). The output layer is then reshaped to take a 2D form, i.e., the 4th and 5th 2D convolution (Conv2D) and max-pooling kernel size of *z* × *z* and stride = 2. We leveraged five convolutional blocks of the ResNeXt-50 model starting from the layer block with filter 128 before the flatten layer, where we freeze the layers from the third block before training. This practice actively discriminates the spatial information within distinct spectral channels without losing any important spectral information. The ResNeXt-50 block (bottleneck layer) further learns deep spatial encoded features when transforming from 3D to 2D before the FCs' layers to significantly condense the input feature maps and accelerate the training speed. Then, the output is downsized (flattened) before assigning it into the FC layers that produce the land-cover class possibilities via a softmax loss layer *l*_0_ expressed as

(8) $$\begin{array}{c} l_{0}=-\frac{1}{p}\sum_{i=1}^{p}\overset{j}{\underset{j=1}{\sum }}\left[r_{ij}\log\left(q_{ij}\right)\right], \end{array}$$

where *j* represents the number of class labels, *p* represents the mini-batch size, and *q*_*i*_ and *r*_*i*_ represent the *i*^th^ label probability distribution vector and the ground truth (GT) label in the mini-batch, respectively. The average is computed on the sum result from the whole mini-batch pixels.

The weights were not significantly changed during the fine-tuning stage, as the ResNeXt-50 model is already good. We employed the Adam optimizer with a learning rate of 0.001 and a weight decay of 1*e* − 06. Usually, the Adam is appropriate for this instead of the SGD optimizer. Whenever the number of training samples is small, it occasionally triggers overfitting. Hence, we adopted early stopping with dropout regularization techniques to combat overfitting and improve generalization error. We used a dropout of 0.50 for IP, PU, SA, and KSC datasets and 0.55 for BS due to the sampled size. We considered the early stopping criterion to quickly stop the training whenever the performance on the validation set detriments and ensures convergence. Therefore, this pattern is factored during the training process to minimize the computation complexity without detrimental classification accuracy. We run each experiment for 100 epochs after estimating the number of components to 75. The batch sizes were set as 25 × 25 × 30 (IP dataset), 25 × 25 × 15 (PU dataset), 25 × 25 × 15 (SA dataset), 25 × 25 × 23 (BS dataset), and 25 × 25 × 15 (KSC dataset), respectively. The PCA technique was used to select the informative bands (i.e., IP = 30, PU = 15, SA = 15, BS = 23, and KSC = 15). We utilized a spatial window size of 25 × 25, similar to the HybridSN model, for an unbiased comparison. See Table 1 for a summary of all layer types, output map dimensions, and the number of parameters used in our proposed model for each dataset.

To solve the quicker convergence of the model, we adopted the ReLUs' activation function. It tends to be faster training convergence than other saturating activation functions. The ReLU also enhances the model's effectiveness to represent complex functions and facilitates optimization, yielding lower training and testing losses and is formulated as

(9) $$\begin{array}{c} f\left(x\right)=\max\left(0,x\right). \end{array}$$

### 3.5. Evaluation Indexes

We use three evaluation metrics, overall accuracy (OA), Kappa coefficient (Kappa), and average accuracy (AA), to estimate the model performance. The OA and AA metrics describe the average exactness of class-wise classification. This helps confirm the precise number of samples correctly classified from the test set. The Kappa coefficient is used as a numerical determination metric to reciprocate information. It helps verify a resilient concurrence based on the ground truth and the classification mapping. See equations (10)–(12) for evaluation indexes.

#### 3.5.1. Kappa Coefficient $\left(\hat{K}\right)$

(10) $$\begin{array}{c} \hat{K}=\frac{P_{0}-P_{c}}{1-P_{c}}, \end{array}$$

where *P*_0_=∑*P*_*ii*_ is the summation of the relative frequency in the diagonal of the actual error and *P*_*c*_=∑*P*_*i*+_*P*_+*j*_ is the relative frequency of random allocation equivalent to the chance of agreement. (“*i*+” and “+*j*”) represents the relative marginal frequencies.

#### 3.5.2. The Overall Accuracy (OA)

(11) $$\begin{array}{c} \text{OA}=\frac{\text{CC}}{T}, \end{array}$$

where CC represents accurately predicted samples in relation to the ground truth. *T* is all samples of either the ground truth or predicted values.

#### 3.5.3. The Average Accuracy (AA)

The average accuracy of our model performance is given by

(12) $$\begin{array}{c} \text{AA}=\frac{1}{C}\sum_{i=1}^{c}x, \end{array}$$

where *c* is the number of classes and *x* indicates the percentage of correctly classified pixels in a single class.

## 4. Experimental and Result Analysis

### 4.1. Data Preprocessing

We processed different publicly available remote sensing datasets [57] to determine the performance of our proposed model. The dataset includes Indian Pines (IP), Pavia University Scene (PU), Salinas Scene (SA), Kennedy Space Center (KSC), and Botswana (BS).  Table 2 summarized the description of each dataset used.

We split the labeled samples randomly into 30% and 10% training set size and 70% and 90% as a test to conduct our experiments, ensuring the inclusion of all classes. Also, we conducted statistical normalization of all the data to zeros and ones-mean (*μ*=0) and unit as the variance (*σ*=1). To measure the volatility of the model, we expressed the classification accuracies using mean (±) standard deviation-based statistics.

We carried a set of experiments to present the effectiveness and superiority of our model. We compared our results with the SOTA, methods such as SVM [53], 2D-CNN [19], 3D-CNN [42], M3D-CNN [54], SSRN [43], and HybridSN [55]. The model obtained a very satisfying performance classification accuracy as compared to the cited methods. In our first experiment, we used 30% of the training samples to determine the best parameters of our model. The results outlined in Tables 3–5 highlight the best classification accuracy for individual classes using categorical_crossentropy as a loss function.

## 5. Results and Discussion

### 5.1. Per-Class Accuracy on the Indian Pines (IP) Dataset

As we can see from Table 3, our proposed model's performance gives the highest score in 10 out of 16 classes on the IP dataset comparing to the methods listed.  Figure 4(a) illustrates the false-color map, Figure 4(b) the reference ground truth map, and Figures 4(c)–4(i) are classification maps for SVM, 2D-CNN, 3D-CNN, M3D-CNN, SSRN, HybridSN, and our proposed model, respectively, on the IP dataset. Our proposed model's quality of the classification map is relatively better than the listed SOTA methods, with a little higher percentage superior to SSRN and HybridSN methods. Our model has a smooth and accurate classification compared to other SOTA models. See red “+” on the class labels such as alfalfa, corn-no till, corn, grass-pasture, grass-trees, grass-pasture-mowed, soybean-min till, soybean-clean, wheat, buildings-grass-trees-drives, and stone-steel-towers.  Figure 5 shows our proposed model's accuracy and loss convergence with 100 epochs on a 30% train set of the IP dataset.

### 5.2. Per-Class Accuracy on Pavia University Scene (PU) Dataset

Table 4 presents the classification results for the PU dataset. In terms of class accuracy, the class “Shadows” happens to be the most challenging to be correctly classified. Our model still exhibits the best accuracy for this class.

Figure 6(a) portrays the false-color map, Figure 6(b) the reference ground truth map, and Figures 6(c)–6(i) are classification maps for the PU dataset employing SVM, 2D-CNN, 3D-CNN, M3D-CNN, SSRN, HybridSN, and our proposed model, respectively. Although the quality of the classification map of SSRN, HybridSN is better, and our model comparatively has a small percentage increment superior to SSRN and HybridSN methods. Our model has a precise and accurate classification compared to other methods with red “+” on the trees, bare soil, and self-blocking bricks class labels. Also, see Figure 7 for the accuracy and loss convergence of our proposed model for 100 epochs on the PU dataset, demonstrating computational effectiveness with significant convergence at approximately 30 epochs.

### 5.3. Per-Class Accuracy on the Salinas Scene (SA) Dataset

The classification accuracy for the SA dataset is shown in Table 5. We trained the model by adopting the Adam optimizer and maintaining a learning rate of 0.001 and 0.50 dropout. It outperforms all other methods, and it has the same performance as HybridSN, however, better in computational efficiency.

Figure 8(a) portrays the false-color map, Figure 8(b) the reference ground truth map, and Figures 8(c)–8(i) are classification maps for the SA dataset using SVM, 2D-CNN, 3D-CNN, M3D-CNN, SSRN, HybridSN, and our proposed model, respectively. The quality of the classification map is still comparatively better with our model, with a significant percentage surpassing the SSRN and HybridSN models. Also, our model has a distinct and correct classification with no ambiguity in the class label. Other SOTA methods with red “+” on the class labels depict misclassification. These labels are Fallow_rough_plow, Corn_senesced_green_weeds, and Vinyard_untrained.  Figure 9 gives the accuracy and loss convergence of the train set on the SA dataset with 100 epochs of our proposed model. The model converges at approximately 40 epochs, confirming that our model delivers high computation efficiency using 30% of the train set.

With 30% train data, we can conclude that our model outperformed other SOTA models. Notably, we compared our model with the HybridSN [46] method using 30% of the available labeled samples in the KSC and BS datasets as the training set.  Table 6 records the result of per-class classification accuracy for the BS dataset. Several works from the literature have not published any results on the BS dataset. However, running the HybridSN [46] model on the BS dataset for comparison confirms that our model performs better on the BS dataset. The BS dataset requires further study on the application of HSI models as it is characterized by low spatial resolution multispectral satellite images.  Table 7 shows the per-class accuracy achieved on 30% of the training set on the KSC dataset. The bold points emphasize the best of our model compared to the HybridSN model.

As shown in Figure 10, our model's training accuracy and loss convergence after 100 epochs engaging 30% of the BS data as a training set. The model converges at almost 50 epochs, verifying quick feature learning of our model.

Table 8 presents the overall accuracy performance regarding OA, Kappa, and AA for classic classifiers and deep neural network models. Our model achieves competing accuracy across the three datasets (IP, PU, and SA), maintaining a minimum standard deviation across all the experiments consecutively. This is due to a sequential representation of spectral-spatial 3D-CNN and a spatial 2D-CNN, succeeded by ResNeXt-50 for feature extraction.

From Table 8, our model outperforms SVM in terms of OA, Kappa, and AA with 14.55, 16.73, and 20.73 percentage points, respectively, on the IP dataset. Additionally, it yielded better classification results than the 2D-CNN, 3D-CNN, M3D-CNN, SSRN, and HybridSN with an OA, Kappa, and AA accuracies of 99.85%, 99.83%, and 99.76%, respectively. Figures 11(a)–11(c) sequentially represent an absolute confusion matrix highlighting the proposed model's performance on 30% training samples of the IP, UP, and SA datasets. We recognize that relatively great diagonal values with different colors are situated across the central diagonal of the entire matrices. This signifies that our model significantly decreases the misclassifications of class labels, with many of the classes precisely predicted, producing a more related map regarding the ground truth.

Table 9 demonstrates the results of our proposed model with various SOTA methods on IP, PU, and SA with 10% of the training set. Our model achieves higher classification accuracy in all considered HSI scenes. The overall accuracy (OA), respectively, mounted to 98.78%, 99.80%, and 99.99% on IP, PU, and SA datasets. Hence, proving our proposed model is somewhat better to the SOTA methods in nearly all states, while maintaining the least standard deviation.

Figures 12–14 emphasizes the training accuracy and loss for our proposed model, and Figure 15 illustrates the confusion matrix of the three datasets, i.e., IP, PU, and SA.

Table 10 presents the execution time on the IP, PU, and SA datasets with spectral-spatial SOTA methods. The execution time is based on the GPU computational training time (m) and testing time (s). We can conclude that our model outperforms the other spectral-spatial models in training and test time. This is due to early stopping, accuracy monitoring, and adopted regularization technique during the training process that helps minimize computational complexity, while steadily maintaining classification performance.

We ran this on MacBook Pro (Retina, macOS Catalina, and processor: 2.3 GHz Quad-Core Intel Core i7, 8 GB 1600 MHz DDR3-NVIDIA GeForce GT 650M (Memory), and Software: Python and Google Colaboratory ltd., with 1 GPU acceleration mode and 25.7 GB RAM.

## 6. Conclusion

This work extends the HybridSN model by proposing a 3D-2D convolutional neural network and transfer learning model for the HSI classification. We introduced a bottleneck layer (ResNeXt-50) in our model to drastically decrease the number of parameters. This helps minimize the computational time than the HybridSN model, while steadily maintaining classification performance. To combat overfitting, we employ early stopping with dropout regularization techniques. The advantage of our 3D-2D convolutional neural network and transfer learning model is the ability to perform highly in a spectral-spatial way. Experiments with five diverse HSI datasets prove that our proposed model did exceptionally well and showed effectiveness. It outperforms the SOTA approaches; hence, it confirms more understanding of the 3D spectral-spatial HSI classification. However, we only trained a few datasets on our model. We recommend future works to consider additional datasets for training and testing our model and implementing them to deep learning methods in HSI classification.

## Figures and Tables

**Figure 1:** General diagram of our proposed method for hyperspectral image classification.

**Figure 2:** Proposed 3D-2D convolutional neural network and transfer learning model architecture.

**Figure 3:** Spectral-spatial hyperspectral image preprocessing through principal component analysis (PCA) for data dimensionality reduction of five datasets.

**Figure 4:** The Indian Pines (IP) hyperspectral data, (a) is the false-color composite, (b) the reference ground truth (GT) map, and (c)–(i) are the classification maps for SVM, 2D-CNN, 3D-CNN, M3D-CNN, SSRN, HybridSN, and our proposed model, respectively. We indicate the classes that were not classified correctly with “+.”

**Figure 5:** The model accuracy and loss convergence on 30% of the train set on the Indian Pines (IP) dataset.

**Figure 6:** The Pavia University (PU) hyperspectral data, (a) is the false-color composite, (b) the reference ground truth (GT) map, and (c)–(i) the comparison classification maps for SVM, 2D-CNN, 3D-CNN, M3D-CNN, SSRN, HybridSN, and our proposed model, respectively. The classes that were not classified correctly are indicated with “+.”

**Figure 7:** The model accuracy and loss convergence on 30% of the train set on the Pavia University (PU) dataset.

**Figure 8:** The Salinas Scene (SA) hyperspectral data, (a) is the false-color composite (b) the reference ground truth (GT) map, and (c)–(i) are the comparison classification maps for SVM, 2D-CNN, 3D-CNN, M3D-CNN, SSRN, HybridSN, and our proposed model, respectively. The classes that were not classified correctly are indicated with the red “+” symbol.

**Figure 9:** The model accuracy and loss convergence on 30% of the train set on the Salinas Scene (SA) dataset.

**Figure 10:** The model accuracy and loss convergence on 30% of the train set on the BS dataset.

**Figure 11:** The confusion matrices of the (a) Indian Pines (IP), (b) Pavia University (PU), and (c) Salinas Scene (SA) hyperspectral data for the 30% train set.

**Figure 12:** The model accuracy and loss convergence for the Indian Pines (IP) dataset with a 10% train data.

**Figure 13:** The model accuracy and loss convergence for the Pavia University (PU) dataset with a 10% train data.

**Figure 14:** The model accuracy and loss convergence for the Salinas Scene (SA) dataset with a 10% train data.

**Figure 15:** The confusion matrices of the (a) Indian Pines (IP), (b) Pavia University (PU), and (c) Salinas Scene (SA) hyperspectral data for the 10% train set.

**Algorithm 1:** Principal component analysis.

**Table 1:** The illustration of the layer-wise summary of our proposed a 3D-2D convolutional neural network and transfer learning model with a window size of 25 × 25. The last layer of our model covers the used dataset, i.e., the Pavia University Scene (PU), Salinas's Scene (SA), Indian Pines (IP), Botswana (BS), and Kennedy Space Center (KSC) datasets.

Layer (type)	No. filters	Kernel size	Output shape	Parameters				
				IP	PU	SA	KSC	BS
Conv_1	8	3 × 3 × 7	25 × 25 × 15 × 8	512	512	512	512	512
3D_MaxPooling	8	2 × 2 × 2	24 × 24 × 14 × 8	0	0	0	0	0
Conv_2	16	3 × 3 × 5	24 × 24 × 14 × 16	5,776	5,776	5,776	5,776	5,776
3D_MaxPooling	16	2 × 2 × 2	23 × 23 × 13 × 16	0	0	0	0	0
Conv-3	32	3 × 3 × 3	23 × 23 × 13 × 32	13,856	138,56	13,856	13,856	13,856
3D_MaxPooling	32	2 × 2 × 2	11 × 11 × 6 × 32	0	0	0	0	0
Reshape	32		11 × 11 × 192/448/192/160	0	0	0	0	0
2D-Conv	64	3 × 3	11 × 11 × 64	110,656	258,112	110,656	92224	92,224
2D-MaxPooling	64	3 × 3	5 × 5 × 64	0	0	0	0	0
Bottleneck	24	1 × 1	5 × 5 × 24	1560	1560	1560	1560	1560
Flatten			600	0	0	0	0	0
Dense_1			256	153,856	153,856	153,856	153,856	153,856
Dropout_1			256	0	0	0	0	0
Dense_2			128	32,896	32,896	32,896	32,896	32,896
Dropout_2			128	0	0	0	0	0
Dense_3			16/9/16/13/14	1,161	2,064	2,064	1,677	1,806
**Total trainable parameters**				**320,273**	**468,632**	**321,176**	**219357**	**320,789**
Dropout				0.5	0.5	0.5	0.5	0.55
Learning rate (lr)				0.001	0.001	0.001	0.001	0.001
Epoch				100	100	100	100	100
Weight decay				1*e* − 06	1*e* − 06	1*e* − 06	1*e* − 06	1*e* − 06
Ncomponents				75	75	75	75	75
Window size				25 × 25	25 × 25	25 × 25	25 × 25	25 × 25

**Table 2:** Summary of hyperspectral image datasets used in our experimentation.

Dataset name	Publication year	Mode	Data collection location	Pixels	Spatial dimension (pixels)	Spectral bands	Wavelength range (nm)	Labels	Classes	Spatial resolution (m)
IP	1992	NASA AVIRIS	North Western Indiana	21025	145 × 145	220	400–2500	10249	16	20

PU	2001	ROSIS-03 sensor	Northern, Italy	991040	610 × 610	115	430–860	50,232	9	1.3

SA	1998	NASA AVIRIS	Salinas Valley, California	111104	512 × 217	224	360–2500	54129	16	3.7

KSC	1996	NASA AVIRIS	Florida	314368	512 × 614	224	400–2500	5211	13	18

BS	2001–2004	NASA EO-1	Okavango Delta, Botswana	377856	1496 × 256	242	400–2500	3248	14	30

**Table 3:** Classification and analysis result of per-class accuracy on the Indian Pines (IP) Scene.

#	Class labels	Train/test	SVM	2D-CNN	3D-CNN	M3D-CNN	SSRN	HybridSN	Proposed
C1	Alfalfa	14/32	82.2	75	79.23	97.03	97.82	99.38	**100**
C2	Corn-notill	428/1000	73.82	81.4	88.6	97.9	99.17	99.58	**99.8**
C3	Corn-mintill	249/581	82.15	87.6	85.81	92.41	99.53	99.66	99.31
C4	Corn	71/166	77.12	62.04	90.53	93.25	97.79	99.88	**100**
C5	Grass-pasture	145/338	73.66	92.3	96.11	95	99.24	99.53	**100**
C6	Grass-trees	219/511	93.4	99.21	98.43	99.74	99.51	99.96	**100**
C7	Grass-pasture-mowed	8/20	96.21	75	92.36	100	98.7	99	**100**
C8	Hay-windrowed	143/335	85.72	100	98.51	99.99	99.85	100	100
C9	Oats	6/14	97.38	64.28	88.9	96.61	98.5	100	99.86
C10	Soybean-notill	292/680	71.01	82.79	87.72	96.32	98.74	99.56	**99.71**
C11	Soybean-mintill	736/1719	76.5	91.27	91.42	97.13	99.3	99.84	**99.94**
C12	Soybean-clean	178/415	83.9	82.89	90.04	97.16	98.43	99.52	**99.76**
C13	Wheat	62/143	83.56	99.3	99	99.6	100	99.86	**100**
C14	Woods	379/886	98.63	98.87	97.95	98.42	99.31	100	100
C15	Buildings-grass-trees-drives	116/270	94.21	86.29	82.57	83.31	99.2	99.85	**100**
C16	Stone-steel-towers	28/65	69.63	100	98.51	100	97.82	98.46	**100**

**Table 4:** Classification and analysis result of per-class accuracy on Pavia University Scene (PU) dataset.

*#*	Class labels	Train/test	SVM	2D-CNN	3D-CNN	M3D-CN	SSRN	HybridSN	Proposed
C1	Asphalt	1989/4642	94.72	98.51	98.4	98.31	100	100	100
C2	Meadows	5594/13055	97.15	99.54	96.91	96.1	99.87	100	100
C3	Gravel	630/1469	82.73	84.62	97.05	96.34	100	100	100
C4	Trees	919/2145	96.82	98.04	98.84	98.82	100	99.84	**99.86**
C5	Painted metal sheets	403/942	99.71	100	100	99.97	100	100	100
C6	Bare soil	1509/3520	90.48	97.1	99.32	99.83	100	100	100
C7	Bitumen	399/931	87.73	95.05	98.92	99.66	100	100	100
C8	Self-blocking bricks	1105/2577	88.29	96.39	98.33	99.23	99.34	99.98	**100**
C9	Shadows	284/663	99.9	99.69	99.9	99.92	100	99.9	99.55

**Table 5:** Classification and analysis result of per-class accuracy on Salinas's Scene (SA) dataset.

#	Classes	Train/test	SVM	2D-CNN	3D-CNN	M3D-CNN	SSRN	HybridSN	Proposed
C1	Brocoli_green_weeds_1	603/1406	99.6	100	98.41	97.5	100	100	100
C2	Brocoli_green_weeds_2	1118/2608	99.82	99.96	100	100	100	100	100
C3	Fallow	593/1383	99.26	99.63	99.23	99.43	100	100	100
C4	Fallow_rough_plow	418/976	99.4	99.28	99.9	99.51	99.89	100	100
C5	Fallow_smooth	803/1875	99.42	99.2	99.43	99.72	100	100	100
C6	Stubble	1188/2771	100	100	99.55	99.23	100	100	100
C7	Celery	1074/2505	99.83	100	99.72	99.45	100	100	100
C8	Grapes_untrained	3381/7890	85.25	93.62	89.75	92.63	100	100	100
C9	Soil_vinyard_develop	1861/4342	99.71	100	99.81	99.7	100	100	100
C10	Corn_senesced_green_weeds	983/2295	97.03	98.82	98.36	97.31	99.91	100	100
C11	Lettuce_romaine_4wk	320/748	98.24	99.73	98.12	98.05	100	100	100
C12	Lettuce_romaine_5wk	578/1349	99.46	100	98.96	98.5	100	100	100
C13	Lettuce_romaine_6wk	275/641	98.77	100	98.93	98.7	100	100	100
C14	Lettuce_romaine_7wk	321/749	97.3	99.86	98.6	98.42	100	100	100
C15	Vinyard_untrained	2180/5088	72.71	91.52	79.31	87.18	99.96	100	100
C16	Vinyard_vertical_trellis	542/1265	99.41	99.92	94.51	91.11	100	100	100

**Table 6:** Classification and analysis result of per-class accuracy on the Botswana (BS) dataset.

#	Class labels	HybridSN	Proposed
C1	Water	100	99.94
C2	Hippo grass	100	100
C3	Floodplain grasses 1	100	100
C4	Floodplain grasses 2	100	100
C5	Reeds 1	94.68	**100**
C6	Riparian	99.47	99.47
C7	Firescar 2	100	100
C8	Island interior	100	99.3
C9	Acacia woodlands	100	100
C10	Acacia shrublands	100	100
C11	Acacia grasslands	100	100
C12	Short mopane	100	100
C13	Mixed mopane	100	100
C14	Exposed soils	96.97	**100**
	**OA**	99.43 ± 0.3	**99.82** ± **0.4**
	**Kappa**	99.38 ± 0.1	**99.81** ± **0.4**
	**AA**	99.36 ± 0.6	**99.84** ± **0.1**

**Table 7:** Classification and analysis result of per-class accuracy on the Kennedy Space Center (KSC) dataset.

*#*	Class label	HybridSN	Proposed
1	Scurb	96.93	**97.08**
2	Willow-swamp	82.19	74.43
3	Cabbage-palm-hammock	86.52	**91.74**
4	Cabbage-palm/oak-hammock	63	**74.45**
5	Slash-pine	95.17	**100**
6	Oak/broadleaf-hammock	83.5	**98.06**
7	Hardwood-swamp	89.36	88.3
8	Graminoid-marsh	91.24	90.46
9	Spartina-marsh	64.32	**64.53**
10	Cattail-marsh	74.18	**95.05**
11	Salt-marsh	100	100
12	Mud-flats	98.01	**100**
13	Water	100	100
	**OA**	88.7	**91.71**
	**Kappa**	87.4	**90.76**
	**AA**	86.49	**90.32**

**Table 8:** The classiﬁcation accuracies (in percentages) on the IP, PU, and SA on our model plus the state-of-the-art methods by a 30% training dataset.

Methods	Datasets								
	IP			PU			SA		
	OA	Kappa	AA	OA	Kappa	AA	OA	Kappa	AA
SVM	85.30 ± 2.8	83.10 ± 3.2	79.03 ± 2.7	94.34 ± 0.2	92.50 ± 0.7	92.98 ± 0.4	92.95 ± 0.3	92.11 ± 0.2	94.60 ± 2.3
2D-CNN	89.48 ± 0.2	87.96 ± 0.5	86.14 ± 0.8	97.86 ± 0.2	97.16 ± 0.5	96.55 ± 0.0	97.38 ± 0.0	97.08 ± 0.1	98.84 ± 0.1
3D-CNN	91.10 ± 0.4	89.98 ± 0.5	91.58 ± 0.2	96.51 ± 0.2	95.51 ± 0.2	97.57 ± 1.3	93.96 ± 0.2	93.32 ± 0.5	97.01 ± 0.6
M3D-CNN	95.32 ± 0.3	99.07 ± 0.3	98.93 ± 0.6	95.76 ± 0.2	94.50 ± 0.2	95.08 ± 1.2	94.79 ± 0.3	94.20 ± 0.2	96.25 ± 0.6
SSRN	99.19 ± 0.3	99.07 ± 0.3	98.93 ± 0.6	99.90 ± 0.0	99.87 ± 0.0	99.91 ± 0.0	99.98 ± 0.1	99.97 ± 0.1	99.97 ± 0.0
HybridSN	99.75 ± 0.1	99.71 ± 0.1	99.63 ± 0.2	99.98 ± 0.0	99.98 ± 0.0	99.97 ± 0.0	100 ± 0.0	100 ± 0.0	100 ± 0.0
**Proposed**	**99.85** ± **0.6**	**99.83** ± **0.2**	**99.76** ± **0.2**	**99.98** ± **0.9**	**99.98** ± **0.4**	**99.97** ± **0.4**	100 ± 0.0	100 ± 0.0	100 ± 0.0

**Table 9:** The classiﬁcation accuracies (in percentages) on the IP, PU, and SA on our model plus the modern classification methods by a 10% training dataset.

Methods	IP			PU			SA		
	OA	Kappa	AA	OA	Kappa	AA	OA	Kappa	AA
2D-CNN	80.27	78.26	68.32	96.63	95.53	94.84	96.34	95.93	94.36
3D-CNN	82.62	79.25	76.51	96.34	94.9	97.03	85	93.2	89.63
M3D-CNN	81.39	81.2	75.22	95.95	93.4	97.52	94.2	93.61	96.66
SSRN	98.45	98.23	86.19	99.62	99.5	99.49	99.64	99.6	99.76
HybridSN	98.39	98.16	98.01	99.72	99.64	99.2	99.98	99.98	99.98
**Proposed**	**98.78**	**98.60**	**98.49**	**99.80**	**99.73**	**99.67**	**99.99**	**99.99**	**99.99**

**Table 10:** Training time (m) and testing (s) on three HSI datasets (IP, PU, and SA).

Data	3D-CNN		HybridSN		Proposed	
	Train (m)	Test (s)	Train (m)	Test (s)	Train (m)	Test (s)
IP	15.2	4.3	14.1	4.8	**9.9**	**3.2**
PU	58.0	10.6	20.3	6.6	**20.2**	**5.3**
SA	74	15.2	25.5	9.0	**24**	**4.9**

## Data Availability

The data that support the findings of this study are openly available in Hyperspectral Remote Sensing Scenes at http://www.ehu.eus/ccwintco/index.php/Hyperspectral_Remote_Sensing_Scenes.
